RETRACTED

# Effects of Laparoscopic Hyperthermic Perfusion Therapy Combined with Adjuvant Treatment of Compound Yew Capsule on Ovarian Blood Flow Parameters and Immune Function in Patients with Ovarian Cancer

**DOI:** 10.1155/2022/9603492

**Published:** 2022-07-13

**Authors:** Mengya Su, Donghui Wang, Ping Huang

**Affiliations:** Department of Gynecology, Cangzhou Central Hospital, Cangzhou, Hebei Province, China

## Abstract

**Objective:**

To determine the effects of laparoscopic hyperthermic perfusion therapy combined with adjuvant compound yew capsules on ovarian blood flow parameters and immune function in patients with ovarian cancer (OC).

**Methods:**

A total of 90 OC patients enrolled in our hospital between January 2019 and January 2020 were randomly distributed into the control (Con group) and experimental group (Exp group) based on the sealed envelope method. The Con group was administered laparoscopic hyperthermic perfusion therapy. On this basis, the Exp group was subjected to compound yew capsules; the ovarian blood flow parameters and immune function indexes were compared between the two groups.

**Results:**

The Exp group was reported to perform better than the Con group regarding ovarian blood flow parameters and immune indexes after treatment (*p* < 0.001).

**Conclusion:**

Laparoscopic hyperthermic perfusion therapy combined with adjuvant compound yew capsules for patients with OC can substantially improve the clinical indexes and immune function. Furthermore, research and adequate promotion are needed to elicit the evidence beyond preclinical studies to understand the intricacies of its implementation.

## 1. Introduction

Ovarian cancer (OC) is a frequently occurring malignant tumor and ranked second after uterine body cancer and cervical cancer [1, 2]. Epithelial cancer and malignant germ cell tumors are common types of OC. The ovarian tumor's symptoms are vague, are not prominent in the early stage, and appear upon progression to the advanced stage. Symptoms include decreased appetite, lower abdominal discomfort, and bloating [3–5]. At present, the pathogenesis of OC has not been fully elucidated. Some scholars believe its etiology is associated with endocrine and fertility factors. If not appropriately diagnosed early, ovarian cancer can be life-threatening and more challenging to treat at later stages [4, 6]. Previously, traditional Chinese medicine (TCM) has been extensively applied as a promising adjunctive drug in the fight against ovarian cancer [7, 8]. For instance, bitter lemon seeds-derived MAP 30 [9] and yew-derived Paclitaxel [10] have recently achieved safe and curative effects against ovarian cancers. The scant research literature and the shortcomings associated with clinical trial design and quality control limit the application of TCM as a viable regimen against ovarian cancer. In recent years, surgery combined with chemotherapy has been the mainstay for clinical treatment of this kind of disease, but the safety concern and reduction in patient ability to resist chemotherapy are the risks associated [11, 12]. The advent of laparoscopic hyperthermic perfusion therapy (LHPT) can improve the efficacy and lower the incidence of adverse reactions through thermal effects. However, it is clinically found that no single treatment method is appropriate. On this basis, the introduction of compound yew capsule adjuvant therapy can effectively improve the clinical indicators of patients [13]. Therefore, this study was designed to explore the influence of LHPT combined with compound yew capsule adjuvant treatment on ovarian blood flow parameters and immune function in patients with OC. Ninety patients treated in our hospital between January 2019 and January 2020 were enrolled as the research objects. The results are reported as follows.

RETRACTED

## 2. Materials and Methods

### 2.1. General Information

A total of 90 OC patients admitted to Cangzhou Central Hospital between January 2019 and January 2020 were distributed into the control group (Con group) and the experimental group (Exp group) based on the sealed envelope method. This study was conducted with approval from the ethics committee of Cangzhou Central Hospital (Approval No. 9297101).

### 2.2. Inclusion Criteria

The inclusion criteria are as follows: ① patients met the diagnostic criteria for OC in *Obstetrics and Gynecology,* in which the diagnosis of OC is based on the patient's personal and family history of gynecologic, breast, and colon cancer, and performed diagnostic tests when necessary [14]; ② patients had a survival time ≥3 months; ③ this study was conducted with approval from the hospital ethics committee (medical scientist, head nurse, clinicians, ethicist, secretary, and medical specialist), and the patient and his family members signed an informed consent form after being apprised of the purpose and process of the study.

### 2.3. Exclusion Criteria

The exclusion criteria are as follows: ① combined with acute and chronic infectious diseases; ② patients who have received antitumor therapy in the past; ③ patients with abnormal heart, lung, liver, and kidney function.

### 2.4. Method

The Con group was administered with LHPT, and ultrasound positioning, routine disinfection, and draping were performed; 1% lidocaine was given to the patients (manufacturer: Shiyao Yinhu Pharmaceutical Co., Ltd.; approval no.: H14024045; specification: 5 ml: 0.1 g) for local anesthesia, the patient's bilateral abdominal cavities were punctured to perform fluid extraction, and the ascites was released through the drainage bag; then, an extracorporeal circulation perfusion machine was used to heat 0.9% saline to a temperature > 42°C. In addition, a puncture needle was used to puncture the abdominal cavity, and the other cavity was used to measure the drainage of ascites. The lavage was continued until the outflow was clear. Finally, a perfusion machine was used to place the indwelling tube on both sides of the abdominal cavity, ensuring the state of one out and one in, and infusion was continued for 60 minutes; after the circulatory treatment was completed, the effusion was drained and the puncture needle was removed. The perfusion was performed 1 time/3 weeks.

RETRACTED

On this basis, the Exp group introduced two pills of compound yew capsules (manufacturer: Chongqing Sino Biopharmaceutical Co., Ltd.; approval no.: Z20026350; specification: 0.3 g^*∗*^12 capsules), 3 times/d.

Both groups underwent 2 months of treatment.

### 2.5. Observation Indicators

A Doppler ultrasound detector (manufacturer: Beijing Kuntaide Medical Technology Co., Ltd.; model: C9) was used to detect the blood volume perfusion index (PI) and the peak systolic velocity (PSV) and resistance index (RI) of both groups before and after therapy.

The immune function indicators of the two groups were compared after therapy. 2 ml of fasting venous blood was collected from both groups of patients. EDTA was used as an anticoagulant, and the flow cytometry (manufacturer: German Partec; model: CyFlow® Ploidy Analyzer) was performed to detect CD4+, CD8+, and CD4+/CD8+ in the *T*-lymphocyte subsets of the patients.

### 2.6. Statistical Analyses

Data analyses were conducted with SPSS20.0 software. The study includes count and measurement data, which were analyzed via the *x*^2^ and *t*-tests. Values of *p* < 0.05 were deemed statistically significant.

## 3. Results

### 3.1. Comparison of General Information

The two groups showed no differences between average age, BMI, pathological type, FIGO staging, and location of residence (*p* > 0.05, Table 1).

### 3.2. Comparison of Ovarian Blood Flow Parameters

After therapy, the ovarian blood flow parameters of the Exp group were notably enhanced as compared to the Con group (*p* < 0.05, Table 2).

### 3.3. Comparison of Immune Indicators

After therapy, the immune indexes of the Exp group were found superior to the Con group (*p* < 0.05, Table 3).

## 4. Discussion

Over the past few years, the incidence of OC has been rising, seriously endangering women's life and health [15]. OC has a high incidence and a high mortality rate. Owing to the insidious symptoms in the early stage, patients with OC are often diagnosed at the advanced stage. A variety of clinical symptoms and difficulty in separating and differentiating between tumor cells prompting the diagnostic treatment approach challenging, which is not conducive to the prognosis of patients [16–18]. At present, the main clinical treatment is surgery combined with chemotherapy. However, because OC is a chemotherapy-sensitive tumor, long-term chemotherapy will not only cause toxic reactions such as immunosuppression but also decrease the immune function of the patient's body. Along with safety concerns, it is also difficult to meet clinical needs [19–21]. Pilot studies have shown that TCM, including MAP 30 and Paclitaxel, has been extensively applied to treat ovarian cancer effectively [8–10, 14]. However, despite extensive clinical research, the clinical efficacy of TCM is still not well understood. Moreover, recent evolution in radiotherapy with the advent of low-dose hyperfractionation, intensity-modulated radiotherapy (IMRT), and stereotactic body radiotherapy (SBRT) [22] have led to unprecedented advances in ovarian cancer and could be reconsidered as the standard treatment modality for this deadly tumor. The possible side effects of toxicity, diarrhea, and successive advancement of systemic therapies have limited radiotherapy's use in treating this disease. It is clinically found that LHPT combined with compound yew capsule adjuvant therapy can substantially improve the patients' clinical indicators, inhibit tumor development, and produce significant clinical effects. Among them, LHPT is to inject chemotherapeutic drugs into the abdominal cavity to directly contact the tumor lesions, reducing the toxic and side effects caused by high-dose intravenous chemotherapy and improving the clinical efficacy of cancerous ascites [23–25]. In addition, heat sensitivity and tolerance of normal human cells are quite different from those of tumor cells. Tumor cells are prone to damage at a temperature between 40°C and 42°C. A large number of tumor cells will be killed upon exposure to this range of temperature. Fortunately, normal cells can tolerate this temperature range, permitting therapy to perform efficiently and effectively against tumors [26–28]. Although laparoscopic hyperthermic perfusion therapy emanates a desirable clinical effect, the single treatment remains unsatisfactory. On this basis, the introduction of compound yew capsules can effectively prolong the patients' survival. Yew capsule such as Paclitaxel is a clear mix of Chinese and Western medicine with both mitogenic and TCM effects. Paclitaxel, a yew-derived (*Taxus brevifolia*) compound, was isolated in 1969 and administered as TCM for relieving cough [29, 30]. Later, one with multiple screening experiments for anticancer activities was approved as a potential anticancer drug by the US Food and Drug Administration in 1992 [31], which is now the first line of treatment against ovarian and breast cancer [32]. Compound yew capsules, as a new type of antimitotic inhibitor, have the effects of dredging collaterals, dispelling lumps, eliminating evils, and strengthening the body. Among them, iron-clad gold can reduce swelling and detoxification and stop bleeding and analgesia; licorice can relieve heart fire, clear heat, and detoxify; and Yew can improve human immunity and suppress tumors; the combination of all these medicines can effectively inhibit the development of the patient's condition. Related studies have found that the blood flow parameters of malignant tumor tissues are characterized by low resistance and high flow rate. Because OC tumors are in a high metabolism state for a long run during the development process, it will cause an increase in blood perfusion and a decrease in vascular resistance. Blood flow parameters are also clinically used as effective indicators for judging OC tumors [33].

RETRACTED

In our study, the Exp group showed notably improved ovarian blood flow parameters than the Con group after therapy induction, indicating that LHPT combined with adjuvant treatment of compound yew capsules can effectively improve the patients' clinical indicators. Moreover, the Exp group showed notably better immune indexes than the Con group after treatment in the study, which was in agreement with the research results of KATO et al. [34], who pointed out that CD4+, CD8+, and CD4+/CD8+ were (38.39 ± 5.41)%, (25.19 ± 3.11)%, and (1.56 ± 0.27), noticeably better than the Con group values (35.16 ± 6.27)%, (29.76 ± 3.73)%, and (1.31 ± 0.18). It fully demonstrates that LHPT combined with compound yew capsule treatment can enhance the patient's immunity by elevating the abovementioned immune cells by increasing the expression of both MHC-I and PD-L1, as reported previously [32].

Previously, various combinational therapies have been administered with fruitful results. For instance, chemotherapy has been used as adjuvant therapy in combination with radiation therapy [35], chemotherapy [36], antiangiogenesis drugs [37], and poly-ADP ribose polymerase inhibitors (PARPi) [38], yielding significant results including enhanced antitumor activities against ovarian cancer and increased survival time. The present study's findings concord with the previously mentioned combination therapies.

RETRACTED

The preliminary limitation of the current study was the clinical trials endorsed in the Chinese population without taking other populations into consideration. This result fails to figure out the intricacies of the novel treatment strategy in different populations, thus limiting the reliability and accuracy of the conclusion. Another limitation of the study was selecting a small sample size. Furthermore, research is needed to validate the findings of the present study by endorsing large-scale clinical trials.

In summary, the combination of LHPT and compound yew capsules in patients with OC can substantially induce a potent CD4+ and CD8+ T-cell-dependent antitumor immune response and enhance the patient's clinical indicators. It deserves promotion and application.

## Figures and Tables

**Table 1:** Comparison of general information of the two groups of patients.

	Experimental group (*n* = 45)	Control group (*n* = 45)	*x* ^2^ or *t*	*p*
Mean age (year)	62.25 ± 3.32	62.33 ± 3.29	0.115	0.909

BMI (kg/m^2^)	26.27 ± 1.59	25.89 ± 1.63	1.119	0.266
Pathological type				

Serous adenocarcinoma	32 (71.11)	30 (66.67)	0.207	0.649
Mucinous adenocarcinoma	7 (15.56)	8 (17.78)	0.080	0.777
Endometrioid carcinoma	6 (13.33)	7 (15.56)	0.089	0.764

FIGO staging			0.051	0.822
III	31 (68.89)	30 (66.67)		
IV	14 (31.11)	15 (33.33)		

Place of residence			0.050	0.822
City	31 (68.89)	30 (66.67)		
Countryside	14 (31.11)	15 (33.33)		

**Table 2:** Comparison of ovarian blood flow parameters between the two groups ($\bar{x}\pm s$).

Groups	*n*	PI		PSV (cm/s)		RI	
		Before treatment	After treatment	Before treatment	After treatment	Before treatment	After treatment
Experimental group	45	0.66 ± 0.05	1.71 ± 0.16	25.88 ± 2.27	16.21 ± 1.52	0.37 ± 0.06	0.79 ± 0.09
Control group	45	0.67 ± 0.04	1.01 ± 0.13	25.86 ± 2.25	20.88 ± 2.02	0.38 ± 0.04	0.42 ± 0.05
*t*		1.048	22.778	0.042	12.392	0.930	24.108
*p*		0.298	<0.001	0.967	<0.001	0.355	<0.001

**Table 3:** Comparison of immune indicators between the two groups ($\bar{x}\pm s$).

Groups	*n*	CD4^+^ (%)		CD8^+^ (%)		CD4^+^/CD8^+^	
		Before treatment	After treatment	Before treatment	After treatment	Before treatment	After treatment
Experimental group	45	36.66 ± 7.15	39.23 ± 5.21	26.88 ± 4.27	23.21 ± 3.85	1.37 ± 0.31	1.79 ± 0.23
Control group	45	36.67 ± 7.21	33.27 ± 6.11	26.86 ± 4.25	30.01 ± 3.93	1.38 ± 0.32	1.42 ± 0.16
*t*		0.007	4.979	0.022	8.291	0.151	8.859
*p*		0.995	<0.001	0.982	<0.001	0.881	<0.001

## Data Availability

All data generated or analyzed during this study are included within this article.
